RETRACTED

# The Early Stage Formation of PI3K-AMPAR GluR2 Subunit Complex Facilitates the Long Term Neuroprotection Induced by Propofol Post-Conditioning in Rats

**DOI:** 10.1371/journal.pone.0065187

**Published:** 2013-06-11

**Authors:** Haiyun Wang, Guolin Wang, Chenxu Wang, Ying Wei, Zhiting Wen, Chunyan Wang, Ai Zhu

**Affiliations:** 1 Department of Anesthesiology, Tianjin Medical University General Hospital, Tianjin Research Institute of Anesthesiology, Tianjin, People's Republic of China; Massachusetts General Hospital, United States of America

## Abstract

Previously, we have shown that the phosphoinositide-3-kinase (PI3K) mediated acute (24 h) post-conditioning neuroprotection induced by propofol. We also found that propofol post-conditioning produced long term neuroprotection and inhibited the internalization of α-amino-3-hydroxy-5-methyl-4-isoxazolepropionic acid (AMPA) receptor GluR2 subunit up to 28 days post middle cerebral artery occlusion (MCAO). However, the relationship between PI3K with AMPA receptor GluR2 subunit trafficking in propofol post-conditioning has never been explored. Here we showed that propofol post-conditioning promoted the binding of PI3K to the C-terminal of AMPA receptor GluR2 subunit and formed a complex within 1 day after transient MCAO. Interestingly, the enhanced activity of PI3K was observed in the hippocampus of post-conditioning rats at day 1 post ischemia, whereas the decrease of AMPA receptor GluR2 subunit internalization was found up to 28 days in the same group. Administration of PI3K selective antagonist wortmannin inhibited the improvement of spatial learning memory and the increase of neurogenesis in the dentate gyrus up to 28 days post ischemia. It also reversed the inhibition of AMPA receptor GluR2 internalization induced by propofol post-conditioning. Together, our data indicated the critical role of PI3K in regulating the long term neuroprotection induced by propofol post-conditioning. Moreover, this role was established by first day activation of PI3K and formation of PI3K-AMPA receptor GluR2 complex, thus stabilized the structure of postsnaptic AMPA receptor and inhibited the internalization of GluR2 subunit during the early stage of propofol post-conditioning.

## Introduction

During the cerebral ischemia, a rise in intracellular calcium ([Ca^2+^]i) is thought to initiate a cascade of events leading to the cell death, including activation of proteases and endonucleases, generation of free radicals that destroy cell membranes by lipid peroxidation, and induction of apoptosis [1]–[6].

Although α-amino-3-hydroxy-5-methyl-4-isoxazolepropionic acid (AMPA) receptors are initially thought to be relatively impermeable to Ca^2+^, it is now clear that there is also AMPA receptor (AMPAR) exhibiting considerable Ca^2+^ permeability. AMPARs containing the GluR2 subunit exhibit low Ca^2+^ permeability, whereas AMPARs lacking GluR2 are much more Ca^2+^ permeable (Cp-AMPARs) [7]–[9]. AMPAR-mediated excitotoxicity is thought to play a critical role in CNS ischemic insults [10], [11]. We have showed that propofol post-conditioning inhibited AMPAR GluR2 subunit internalization in hippocampal neurons and provided neuroprotection to cerebral ischemia/reperfusion (I/R) injury. These effects were sustained to 28 days post-ischemia [12]. Therefore, the maintenance of the surface expression of Ca^2+^-impermeable AMPARs may play the key protective role during cerebral ischemia/reperfusion injury.

RETRACTED

The intracellular signaling pathways, which modulate AMPARs trafficking during such processes, are not fully understood. We have found that propofol post-conditioning displayed the acute (24 h) neuroprotection partly through the phosphorylation of Akt, one of the phosphoinositide-3-kinase (PI3K) effectors [13]. The PI3K/Akt pathway is an attractive target because it has been shown to be involved in the synaptic plasticity, neuroprotection during cerebral ischemia/reperfusion injury [14]–[16]. A previous study showed that a slow, but constant, turnover of phosphatidylinositol-(3,4,5)-trisphosphate (PIP3) at synapses is required for maintaining AMPA receptor clustering and synaptic strength under basal conditions [17]. PIP3 is the product of the reaction catalyzed by Class I PI3K, therefore we hypothesized that keeping the activity of PI3K plays a key role in maintenance the basal structure of the surface AMPARs, thus inhibiting the internalization of AMPAR GluR2 subunit during cerebral ischemia/reperfusion injury.

In this context, we first studied the role of PI3K activation in long term neuroprotection induced by propofol post-conditioning; second, we explored whether the inhibition of PI3K activity can affect the internalization of AMPAR GluR2, and in which pattern them interacted.

## Materials and Methods

Adult male Sprague–Dawley rats (250–280 g) were cared for according to the Guide for the Care and Use of Laboratory Animals. The committee of experimental animals of Tianjin Medical University approved all the surgical procedures. All rats were anesthetized by intraperitoneal injection of Inactin (thiobutabarbital, 100 mg/kg; RBI, Natick, MA) and ventilated with oxygen (35%) and air mixture [12].

### Stroke Model and Grouping

The reversible right side MCAO (60 min) was performed as previous published [13]. Regional cerebral blood flow (CBF) was monitored by laser-Doppler flowmeter (Periflux system 5000; Perimed Inc., Jarfalla, Sweden). The rats that did not show a cerebral blood flow reduction of at least 70% were excluded from the experimental group [18]. One hour after MCAO, the suture was removed to allow reperfusion, confirmed by the increase of CBF at the same area. Polyethylene catheters were inserted into the right femoral artery and vein for blood pressure monitoring, blood gases measurement, and drug administration. Physiological variables (mean arterial blood pressure, temperature, arterial blood gases and plasma glucose) were measured 30 min before ischemia, at the onset of ischemia and 30 min after reperfusion. Body temperature was monitored with a rectal probe and maintained at 37±0.5°C by warming blanket and lamps until the animals showed adequate motor activity.

RETRACTED

All rats were divided randomly into six groups: (i) sham-operated group (n = 65); (ii) Ischemia/Reperfusion (I/R) group: 60 min MCAO followed by reperfusion (n = 60); (iii) propofol Post-cond group: propofol 20 mg/kg/h was infused intravenously with syringe pump (Beijing Slgo Medical Technology Development Co., Ltd., Beijing, China) at the onset of reperfusion for 4 h (n = 64). The other three groups were (iv) Wort + sham-operated group (n = 65); (v) Wort + I/R group (n = 62); (vi) Wort + propofol Post-cond group (n = 64); received wortmannin 0.6 mg/kg intravenously 30 min before sham-operation, MCAO and propofol Post-cond procedures, respectively. In case of sham-operated, I/R, Wort + sham-operated and Wort + I/R group, equivalent dose of saline was administered in the same manner of propofol administration.

### Morris Water Maze Task

On day 9 and 23 after MCAO, rats (n = 8–10/group) were tested for spatial learning memory using Morris Water Maze (MWM) procedure [19], [20]. The MWM training consisted of spatial acquisition and reference memory probe trials. For spatial acquisition, latency (time to reach the platform) and swim speed were recorded with a computerized tracking system (Ethovision 3.0; Noldus Information Technology, Wageningen, the Netherlands). Four trials from four different random start positions at north, east, south, and west were tested daily (each lasted 2 min with 30-s intervals) for 5 days. Rats that failed to find the platform within 2 min were guided and their maximum latency score was recorded as 120 s. At 24 h after the last training day, rats were tested for reference memory. The time period (s) when a rat stayed in the goal quadrant, where the hidden platform was previously located, was recorded and expressed as a percent of time in the 60 s total swimming period. In this study, swimming time and distance within only a 30 cm circular zone around the previous platform, that is, not in the whole quadrant, were recorded [21].

RETRACTED

### Neurogenesis in the Ipsilateral Dentate Gyrus (DG) of Hippocampus

Bromodeoxyuridine (BrdU), a thymidine analog which replaces thymidine in newly synthesized DNA, was used to label endogenous proliferating cells. BrdU (100 mg /kg) was injected intraperitoneally on day 7 to 9 after MCAO. After 28 days, the animals were deeply anesthetized and transcardially perfused with 100 mL normal saline, followed by 50 mL 4% in 0.2 M phosphate buffer. The brains were removed, post-fixed for 24 h in paraformaldehyde–phosphate buffer and placed for 48 h in 30% sucrose. The 33 μm coronal sections of brain were prepared at the level of bregma –3.3±0.2 mm. Ten sections of each brain (n = 4–5 rats/group) with immunofluorescence-double staining were used to calculate the ration between BrdU (anti-BrdU-antibody, Abcam Biotechnology, Cambridge, UK) + neuron-specific nuclear protein (NeuN) (anti-neuron-specific nuclear protein, Chemicon International, Temecula, CA, USA)-positive cells and the total amount of BrdU positive cells. For each section, 50 BrdU positive cells in the ipsilateral dentate gyrus (DG) were analyzed for coexpression of BrdU and NeuN to determine the ratio of newly generated neurons (BrdU + NeuN) to the total amount of newborn cells (BrdU). Positive and negative controls and tests for excluding cross-reactions for the two secondary antibodies were performed.

For the measurement of the dentate gyrus volume, we adapted the method from Engelhard et al. [22]. Briefly, 10 sections (n = 5 rats/group, 40 μm each section) were prepared at the level of bregma –3.3±0.2 mm and stained with hematoxylin and eosin (HE). We measured the dentate gyrus volume of 10 sections for each brain using the Image J software 1.42 (National Institutes of Health, USA). The volume of the dentate gyrus was calculated by multiplying the mean value of the 10 sections with the thickness of one slice (40 μm) and by 10.

### PI3K Activity Measurement

To determine the true activity of PI3K, we preformed a PI3K enzyme-linked immunosorbent assay (ELISA) kit (Cat# K-1000 s, Echelon Biosciences, Salt Lake City, UT, USA) [23], [24]. The rat hippocampus (n = 4–5 rats/group for each time point, 14–15 rats per group) was harvested at day 1, 14 and 28 after MCAO. Saline 0.9% 500 μL was then added and centrifuged for 10 minutes at 12,000 rpm. The upper limpid liquid was aliquoted (∼20 aliquots per rat) and stored at −20°C. We added 25 μL of samples in kinase reaction buffer to an equal volume of 8 μM of phosphatidylinositol-(4,5)-bisphosphate (PIP2) substrate, incubated at 37°C for 2 h. An equal volume of stop solution, containing PIP3 detector and EDTA was then added to stop the reaction. A 100 μL aliquot of this mixture was added to the wells that was coated with PIP3, and then incubated at room temperature for 1 h. Transferred the mixture to corresponding wells of the Detection Plate (K-1001 s) and incubated for 1 h at room temperature, then sealed with the secondary detector (K-SEC1) for 30 min. The reaction was stopped by adding TMB solution (K-TMB1) and read absorbance at 450 nm. The sample values were extrapolated from a standard curve of O.D. vs. known PIP3 concentration, and the activity was expressed as the percentage of control.

RETRACTED

### Detection of AMPA Receptor GluR2 Subunit Internalization and Immunoblotting

Surface and intracellular AMPA receptor GluR2 levels were performed with a protein cross-linking assay [12], [25]. Briefly, On day 1, 14 and 28 after transient MCAO, rats (n = 4–5 rats/group for each time point, 14–15 rats per group) were decapitated, brains were removed rapidly, and the hippocampus was rapidly isolated on an ice-cold platform and chopped into 400 μm slices using a McIllwain tissue chopper (Vibratome, St. Louis, MO). Slices were then incubated with 2 mM bis (sulfosuccinimidyl) suberate (BS^3^; Pierce Biotechnology, Rockford, IL, USA) for 15 min at 4°C. Cross-linking was terminated by 100 mM glycine (10 min at 4°C) and pelleted by brief centrifugation. Samples were aliquoted (∼15 aliquots per rat) and stored at −80°C for further analysis. The protein (30 μg) was separated by SDS/PAGE, transferred to PVDF membranes and probed with primary antibodies for AMPAR subunits GluR2 (Cat# MAB 397, N terminus, 1:1000, Millipore, Billerica, MA) at 4°C overnight. Blots were washed and then incubated with goat anti-mouse IgG secondary antibody conjugated to horseradish peroxidase (1:5000; Millipore). We compared identical amounts of cross-linked and non-cross-linked tissue probed with antibodies to GluR2 to rule out the concern that cross-linking might interfere with immunodetection of the surface band. We used Image J (NIH) to measure the band densities in blinded fashion. T (Total) protein level  =  surface (cross-linked) protein + intercellular (non-cross-linked) protein; S/T ratio  =  surface protein / (surface protein + intercellular protein).

### Coimmunoprecipitation and Western Blotting of PI3K and AMPAR GluR2 Subunit

To determine the relationship between PI3K and AMPAR GluR2 subunit, we used coimmunoprecipitation and immunoblotting assay [26], [27]. At day 1, 14, 28 after MCAO, hippocampus slices (n = 4–5 rats/group for each time point, 14–15 rats per group) were collected and homogenized in lysis buffer with 0.5% Triton X-100, 150 mM NaCl, 5 mM EDTA, and 50 mM Tris supplemented containing protease and phosphatase inhibitors. Total protein were aliquoted (∼5 aliquots per rat) and stored at −80°C. Immunoprecipitations of equivalent protein (100 μg) amounts were performed at 4°C for 4 h by using 1 μg anti-GluR2 antibody (Cat# AB 10529, C terminus, 1:1000, Millipore, Billerica, MA) or an equal amount of control IgG. The antibody protein complexes were captured with protein A/G plus agarose (Santa Cruz Biotechnology). Proteins were eluted from the beads and subjected to SDS-PAGE and immunoblotting for anti-PI3K (Cat# 4292, p85, 1:1000, Cell Signaling, Beverly, MA). Blots were developed using enhanced chemiluminescence detection (Amersham Biosciences). Band intensities were quantified using Image J software 1.42 (National Institutes of Health, USA).

RETRACTED

### Statistical Analyses

Data are presented as mean ± SEM. Statistical calculations were performed in SPSS 16.0 (SPSS Science, Inc., Chicago, IL, USA). Probe test data of MWM and neurogenesis were analyzed by one-way ANOVA and followed by post-hoc Turkey test. The latency of MWM and physiological parameters were analyzed using a four factors (ischemia × propofol × wortmannin × time) repeated measures ANOVA, followed by post-hoc Turkey test. Separate univariate analyses of ELISA and Western blot data were performed with respect to ischemia/reperfusion injury exposure, propofol post-conditioning, wortmannin administration and days of recovery, followed by post-hoc Turkey test. A value of *P*<0.05 was considered as statistically significant.

## Results

### Physiological Variables

All rats were anesthetized with Inactin (thiobutabarbital, 100 mg/kg) at the beginning of our experiment, and the long-lasting effect of Inactin maybe the reason for no or little movement in rats. The animals receiving the 20 mg/kg/h dose of propofol were heavily sedated with little or no movement and did not show any response to the withdrawal reflex resulting from pinching the hind paw. No statistical differences were observed in physiological parameters (mean arterial blood pressure, temperature, arterial blood gases and plasma glucose) between the groups at each time point (data not shown). Rats weighted from 250 to 280 g, with a median weight of 263.4 g. The rectal temperature was maintained at 37±0.5°C by warming blanket and lamps. Major bleeding was observed in four rats, which were removed from the study.

### Spatial Memory Outcome

In the two sessions of training (day 9 to 13 and day 23 to 27, Figure 1A and B), rats in propofol Post-cond group required less time to find the platform than those in I/R group (from day 10 to 13, *P*<0.0001; from day 23 to 27, *P*<0.0001, respectively), although they spent more time than those in sham-operated group (from day 10 to 12, *P*<0.0001; from day 24 to 26, *P*<0.0001; *P* = 0.012 at day 13, *P* = 0.001 at day 23 and *P* = 0.014 at day 27, respectively). Pretreatment of wortmannin, which is a selective PI3K inhibitor, increased the escape latencies (*P* = 0.002 at day 10; *P*<0.0001 vs. propofol Post-cond group at the other days). As expected, the latency (the time to reach platform) and path length were significantly shortened during the two trials of 5-day acquisition period, suggesting that spatial acquisition had developed. Although the analysis of escape latency revealed significant differences between groups, there were no significant differences in the swimming speed between these groups (averaged 0.25±0.04 m/s).

RETRACTED

**Figure 1:** Propofol post-conditioning enhanced the spatial learning memory ability of rats after transient MCAO, whereas selective PI3K antagonist wortmannin decreased it. (**A**) Escape latency in the first session from day 9 to 13. (**B**) Escape latency in the second session from day 23 to 27. (**C**) Time in the target quadrant in probe trials (day 14 and 28). Data are expressed as mean ± SEM (n = 8–10/group), *P<0.05, **P<0.01. Sham, sham-operated group; I/R, I/R group; Pro, propofol Post-cond group; W + sham, Wort + sham-operated group; W + I/R, Wort + I/R group; W + Pro, Wort + propofol Post-cond group.

In the two sessions (14 and 28 days after reperfusion) of probe test, rats in propofol Post-cond group spent significantly more time than those of I/R group in the quadrant where the platform had been (32.0±1.6 vs. 21.5±2.5, *P*<0.0001 at day 14; 37.8±1.8 vs. 32.5±2.1, *P* = 0.004 at day 28), but the time was decreased by administration of wortmannin (25.2±1.9 vs. 32.0±1.6, *P* = 0.003 vs. propofol Post-cond group at day 14; 25.2±1.9 vs. 21.5±2.5, *P* = 0.001 vs. I/R group at day 14; 31.4±3.4 vs. 37.8±1.8, *P*<0.0001 vs. propofol Post-cond group at day 28; 31.4±3.4 vs. 32.5±2.1, *P* = 0.515 vs. I/R group at day 28; Figure 1C).

### Neurogenesis in the Ipsilateral DG of Hippocampus

The newly generated neurons in the ipsilateral DG after 28 days of survival are shown in Figure 2A and B. Twenty-eight days after transient MCAO, the amount of BrdU + NeuN positive neurons increased 1.5 folds in the DG of I/R group as compared with that of sham-operated group (252.3±22.1%, *P*<0.0001). Propofol administration for 4 h from the beginning of reperfusion stimulated neurogenesis in the ipsilateral DG as compared with that of I/R group (434.0±19.5% vs. 252.3±22.1%, *P*<0.0001). Wortmannin eliminated the stimulation of neurogenesis induced by I/R insult and propofol post-conditioning (for Wort + I/R group: 159.0±10.8% vs. 252.3±22.1%, *P*<0.0001 as compared with I/R group; for Wort + propofol Post-cond group: 267.4±32.9% vs. 434.0±19.5%, *P*<0.0001 as compared with propofol Post-cond group). The average volume of the ipsilateral DG was similar for all groups, independent of the drug usage or cerebral ischemia (Figure 2C).

RETRACTED

**Figure 2:** Effect of propofol post-conditioning and wortmannin on neurogenesis in the DG of hippocampus after transient MCAO. (**A**) BrdU and NeuN immunofluorescence-double staining of new generated neurons in the DG. *Scale bar*: 10 μm. (**B**) Quantification of neurogenesis at day 28 after focal ischemia/reperfusion. (**C**) Quantification of the ipsilateral DG volume in each group. Bar represents mean ± SEM (n = 4–5/group), *P<0.05, **P<0.01. Sham, sham-operated group; I/R, I/R group; Pro, propofol Post-cond group; W + sham, Wort + sham-operated group; W + I/R, Wort + I/R group; W + Pro, Wort + propofol Post-cond group.

### PI3K Activity

PI3K activity was shown in Figure 3. The cerebral ischemia/reperfusion injury inhibited the activity of PI3K at day 1 post MCAO as compared with that of sham-operated group (68.4±4.5% vs. 100.0±4.3%, *P*<0.01), whereas at day 14 and 28, it enhanced the PI3K activity (109.5±6.4%, *P*<0.01 at day 14; 111.2±5.3%, *P* = 0.03 at day 28 vs. sham-operated group, respectively). Propofol post-conditioning increased PI3K activity at day 1 as compared with that of I/R group (187.0±15.2% vs. 68.4±4.5%, *P*<0.01). There was no significant difference between these two groups at day 14 and 28. As compared with sham-operated group, propofol post-conditioning also elevated the activity of PI3K (187.0±15.2% vs. 100.0±4.3%, *P*<0.01 at day 1; 117.0±8.3% vs. 100.0±5.5%, *P*<0.01 at day 14; 111.6±7.4% vs. 100.0±4.3%, *P*<0.05 at day 28, respectively). Administration of PI3K selective inhibitor wortmannin reversed the enhancement of PI3K activity induced by propofol post-conditioning at day 1 (69.4±7.2% vs. 187.0±15.2%, *P*<0.01 vs. propofol post-Cond group, 69.4±7.2% vs. 68.4±4.5%, *P* = 0.842 vs. I/R group), but this effect disappeared at other time points.

**Figure 3:** Effect of propofol post-conditioning and wortmannin on the activation of PI3K after transient MCAO. Bar represents mean±SEM (n = 4–5/group), *P<0.05, **P<0.01. Sham, sham-operated group; I/R, I/R group; Pro, propofol Post-cond group; W + sham, Wort + sham-operated group; W + I/R, Wort + I/R group; W + Pro, Wort + propofol Post-cond group.

### AMPARs GluR2 Subunit Internalization

The GluR2 S/T values in I/R group were significantly reduced as compared with those of sham-operated rats (day 1: 23.0±2.3% vs. 100.0±2.1%; day 14: 36.6±3.3% vs. 100.0±1.4%; day 28: 42.8±5.2% vs. 100.0±1.7%; *P*<0.01 at varies time points), whereas these were increased by propofol post-conditioning (day 1: 66.0±5.0% vs. 23.0±2.3%; day 14: 55.4±3.3% vs. 36.6±3.3%; day 28: 54.4±2.0% vs. 42.8±5.2%; *P*<0.05 vs. I/R group at day 1, 14 and 28 after MCAO, Figure 4A and B), indicating that propofol reversed the internalization of AMPARs GluR2 subunit induced by ischemia/reperfusion injury, and this trend was kept until 28 days after reperfusion. Administration of PI3K selective antagonist wortmannin eliminated the effect of propofol in restricting GluR2-containing AMPARs in the cell surface up to 1 day after transient MCAO (24.6±6.0% vs. 66.0±5.0%, *P*<0.01 vs. propofol Post-con group), whereas this effect disappeared at day 14 and 28 (55.6±3.3% vs. 55.4±3.3%, *P* = 0.913 at day 14; 55.4±6.0% vs. 54.4±2.0%, *P* = 0.505 at day 28 vs. propofol Post-con group, respectively; Figure 4A and B). There was no difference in total subunit protein expression between the six groups on days 1, 14 and 28 after transient MCAO (Figure 4C).

RETRACTED

**Figure 4:** Propofol post-conditioning maintained the surface expression of AMPAR GluR2 subunit during cerebral ischemia/reperfusion injury, whereas wortmannin reversed it on day 1 after transient MCAO. (**A**) Western blot analysis showed BS^3^ cross-linked surface and intracellular pools of AMPAR GluR2 subunit at day 1, 14 and 28 after reperfusion. (**B**) Quantification of surface/total GluR2 subunit expression after reperfusion. (**C**) Quantification of total GluR2 subunit expression. Bar represents mean ± SEM (n = 4–5/group), *P<0.05, **P<0.01. Sham, sham-operated group; I/R, I/R group; Pro, propofol Post-cond group; W + sham, Wort + sham-operated group; W + I/R, Wort + I/R group; W + Pro, Wort + propofol Post-cond group.

### Coimmunoprecipitation and Immunoblotting of PI3K and AMPAR GluR2 subunit

As shown in Figure 5A and B, the cerebral ischemia/reperfusion injury caused a significant reduction of PI3K p85 subunit which bound to C-terminal of AMPARs GluR2 (76.8±5.8% vs. 100.0±4.8%, *P*<0.01 vs. sham-operated) at day 1 after MCAO. Rats in propofol Post-cond group showed an increase in bound PI3K (180.4±5.1% vs. 100.0±4.8%, *P*<0.01 vs. sham-operated; 180.4±5.1% vs. 76.8±5.8%, *P*<0.01 vs. I/R group, *P*<0.001, respectively) at day 1. Wortmannin inhibited the binding of PI3K with C-terminal of GluR2 subunit in the other three groups (for Wort + sham-operated group: 91.6±6.0% of sham-operated group, *P*>0.05; for Wort + I/R group: 70.9±4.6% vs. 76.8±5.8%, *P*>0.05 as compared with I/R; for Wort + propofol Post-cond group: 120.4±1.9% vs. 180.4±5.1%, *P*<0.01 as compared with propofol Post-cond group). We can not detect such interaction between PI3K and AMPAR GluR2 subunit at day 14 and 28 after MCAO.

RETRACTED

**Figure 5:** Propofol promoted the formation of PI3K-AMPAR GluR2 complex in the early stage (1 day) after transient MCAO, whereas wortmannin inhibited it. (**A**) Immunoprecipitation and immunoblotting assays showed PI3K-AMPARs GluR2 binding after transient MCAO. (**B**) Quantification of the binding of PI3K to the C-terminal of AMPAR GluR2 subunit at day 1, 14 and 28 after MCAO. Bar represents mean ± SEM (n = 4–5/group), *P<0.05, **P<0.01. Sham, sham-operated group; I/R, I/R group; Pro, propofol Post-cond group; W + sham, Wort + sham-operated group; W + I/R, Wort + I/R group; W + Pro, Wort + propofol Post-cond group.

In the present study, we reported an important role of stimulation and maintenance the activity of PI3K during the early stage (24 h) of propofol post-conditioning, which could improve MWM performance, increase neurogenesis in the ipsilateral DG of hippocampus and inhibit the internalization of AMPAR GluR2 subunit (Ca^2+^ impermeable AMPARs) up to 28 days for cerebral ischemia/reperfusion injury rats. Our results supported this finding by administration of selective PI3K antagonist wortmannin, which reversed the improvement of spatial learning memory, the increase of neurogenesis and the inhibition of GluR2 internalization induced by propofol post-conditioning after transient MCAO. We also detected the formation of intracellular PI3K-AMPAR GluR2 subunit complex at the acute phrase of PI3K activation, indicating a critical protective PI3K-AMPAR GluR2 pathway which mediates propofol induced post-conditioning.

## Discussion

In the adult brain, the persistent neuronal production suggested a potential ability for self-repair after injury [28], [29], especially following ischemic brain injury [30]. After ischemia, the proliferation of progenitors was upregulated several fold, and roughly half of postischemic precursors acquired neuronal phenotype in the granule cell layer of DG, while a few became astrocytes in CA4 sector [31]. About 80% of the initially proliferated cells disappear within 4 wk post ischemia, only the long-term surviving neurons may contribute to postischemia recovery [32]. This is the reason we chose 28 days to check the generation of neurons in the DG of hippocampus. In the current study, we found that cerebral ischemia/reperfusion injury stimulated neurogenesis in the ipsilateral DG to 252.3% of sham-operated group. Propofol post-conditioning promoted the increase of new neurons from 252.3% to 434.0%, whereas pretreatment of the selective PI3K antagonist wortmannin eliminated the stimulation of neurogenesis induced by ischemic insult (from 252.3±22.1% to 159.0±10.8%) and propofol post-conditioning (from 434.0±19.5% to 267.4±32.9%). We also assessed the learning ability and spatial memory by MWM, and found that the improved spatial acquisition were seen in propofol-treated rats, suggesting that propofol post-conditioning induced increases in post stroke neurogenesis may contribute to post stroke recovery. In our experiments, we could not detect the statistical differences in physiological parameters (mean arterial blood pressure, temperature, arterial blood gases and plasma glucose) between the groups at each time point. We still found that the blood pressure of rats in propofol used groups was a little bit lower than the other groups. The decreased blood pressure may negate the neuroprotection induced by propofol post-conditioning.

RETRACTED

Currently several molecular regulatory pathways are known to be involved in the neuroprotective mechanisms of ischemic post-conditioning, as it increased the expression of glutamine synthetase [33] and glutamate transporter-1 [34] in global ischemia; promoted the opening of mitochondrial potassium ATP-dependent channel (mitoK(ATP)), thus inhibited the opening of mitochondrial permeability transition pore (MPTP) in focal cerebral ischemia [35]. PI3K survival signaling pathway supports cell survival [36], including its role in blocking neuronal death after stroke [37], [38]. Previously, we observed that propofol post-conditioning established acute (24 h) neuroprotection partly through the activation of Akt, a central effector in the PI3K pathway [13]. However, the role of PI3K/Akt pathway in modulating the long term effect of propofol post-conditionig has never been explored and the phosphorylated level of Akt can not totally represent the activation of PI3K [39]. In the present study, we investigated the activity of PI3K with the competitive ELISA method which measures the catalyzed production of PIP3 produced by activated PI3K [23], [24]. We found that cerebral ischemia/reperfusion decreased PI3K activity from baseline (sham-operated group, 100.0%±4.3%) to 68.4%±4.5% (*P*<0.01), whereas propofol post-conditioning increased it to 187.0%±15.2% at day 1. At day 14 and 28, the activity of PI3K declined almost to the baseline level (117.7%±8.3% at day 14, 111.6%±7.4% at day 28), with propofol 20 mg/kg/h post-conditioning exposure. The selective PI3K antagonist wortmannin exposure inhibited the expected increase in PI3K activity following propofol post-conditioning at 1 day after transient MCAO in rat hippocampus, from the increase of 187.0%±15.2% dropped to 69.4%±7.2% of baseline. However, such effect disappeared at day 14 and 28 due to the half-life of of wortmannin was 57.8 h in PBS [40], [41].

RETRACTED

AMPARs mediate fast synaptic transmission at excitatory synapses in the central nervous system (CNS) and are heteromeric complexes composed of glutamate receptor subunit 1–4 (GluR1-GluR4) [42], [43]. Of these, the GluR2 subunit plays a crucial role in controlling the calcium permeability of AMPA receptors. GluR2 mRNA ordinarily undergoes post-transcriptional editing so that the expressed protein contains a positively-charged arginine in place of the gene-encoded glutamate at a critical position in the M2 membrane loop that forms the lining of the AMPA receptor's pore [44]. Therefore, GluR2-lacking AMPAR-mediated excitotoxicity is thought to play a critical role in CNS ischemic insults [10], [45]. Our previous study showed that AMPAR GluR2 subunit in hippocampal neurons redistributed to the cell surface during propofol post-conditioning and this effect sustained to 28 days post-ischemia. However, when ischemic rats were challenged with saline, the AMPARs GluR2 subunit S/T ratio decreased, indicating a reduction in the cell surface expression. What are the intracellular signaling pathways that produce either net AMPAR insertion or internalization, thereby dictating the expression of these two opposing forms of AMPAR-dependent synaptic plasticity? A recent study showed that continuous synthesis and availability of PIP3 at the postsynaptic terminal was necessary for sustaining synaptic function in rat hippocampal neurons. This requirement was specific for synaptic, but not extrasynaptic, AMPA receptors [17]. As PIP3 is the catalyzed production of PI3K, we speculate that the activition of PI3K is necessary for the maintenance of AMPARs GluR2 subunit expression at postsynaptic membrane. Interestingly, we found here, the administration of selective PI3K antagonist wortmannin suppressed the AMPARs GluR2 subunit S/T ratio, thus reversed the inhibition of GluR2 internalization induced by propofol post-condittioning during the first day after cerebral ischemia/reperfusion injury, such effect of wortmannin disappeared at day 14 and 28 after transient MCAO duo to its metabolism *in vivo* [37], [38].

However, the pattern in which PI3K communicated with AMPARs GluR2 is largely unknown. The p85 regulatory subunit of PI3K contains multiple protein-protein interaction motifs [46]. Therefore, we hypothesize that this subunit directly binds to regions of the C-terminal of GluR2, and regulates its trafficking. Consistent with this hypothesis, we found that C-terminal of GluR2 antibody could specifically precipitate PI3K p85 subunit of hippocampal lysate using a coimmunoprecipitation assay (Figure 5A). We further found that ischemia/reperfusion injury decreased the formation of such PI3K-GluR2 complex, whereas propofol post-conditioning increased it. Furthermore, adding wortmannin significantly suppressed the elevated formation of this complex induced by propofol post-conditioning. In our present study, such changes of the PI3K-GluR2 complex could only be detected in hippocampus at day 1 after transient MCAO, suggesting that PI3K regulated the internalization of AMPARs GluR2 through the formation of intracellular complex with C-terminal of GluR2 at the early stage of propofol post-conditioning. However, in the post-conditioning group, the PI3K activity declined to the baseline at 14 and 28 days post ischemia, whereas the inhibition of AMPARs GluR2 subunit internalization sustained to 28 days implied that in addition to PI3K, there was other alternate pathways which could maintain the recruiting of AMPARs GluR2 to cellular membranes, thus minimize delayed cerebral injury during propofol post-conditioning. Another attractive scenario is that, in spit of the surface and synaptic GluR2 distribution altered, the total protein levels of GluR2 subunit were unaltered in hippocampal neurons between 6 groups at all times examined. The above results indicated that during ischemic insults, facts of GluR2-lacking AMPARs to be delivered and GluR2-containing AMPARs must be removed, were consistent with a role for placeholders or “slots” that specify (delimit) AMPAR number at synaptic sites [47]. Although the molecular identify of the slots is unknown, receptor-binding or scaffolding proteins such as stargazin are thought to participate in slot formation [48].

RETRACTED

The activation of PI3K and the formation of PI3K-AMPAR GluR2 complex in propofol post-conditioning group within the first day post ischemia, whereas the improvement of spatial learning memory, enhanced neurogenesis in the ipsilateral DG and inhibited the internalization of AMPAR GluR2 subunit (Ca^2+^ impermeable AMPARs) up to 28 days in the same group. All these observations suggested that alternative pathways may regulate the long term neuroprotection of propofol post-conditioning after the function of PI3K disappeared in a PI3K-independent manner [39], [49].

In conclusion, we presently showed that propofol post-conditioning (20 mg/ kg/ h infused at the onset of reperfusion for 4 h) provided long term neuroprotection through enhancing the activity of PI3K, thereby promoted the binding of PI3K to the C-terminal of AMPA receptor GluR2 subunit within 1 day after transient MCAO, thus stabilized the structure of postsynaptic AMPA receptor and decreased the internalization of AMPA receptor GluR2 subunit during cerebral ischemia/reperfusion injury. Our data indicated the important role of maintenance PI3K activity in regulating the long term (28 days post ischemia) neuroprotection induced by propofol post-conditioning. Moreover, our study also showed that the decrease of AMPA receptor GluR2 subunit internalization, the improvement of spatial learning memory ability and the increase of neurogenesis in the ipsilateral DG of hippocampus up to 28 days in the same group, indicating that when the effect of PI3K disappeared, there will be other upstream what could provide sustained neuroprotection for propofol post-conditioning.
